This article has been retracted.

# Hemichorea: A Rare Neurological Complication of Diabetes Mellitus

**DOI:** 10.7759/cureus.21131

**Published:** 2022-01-11

**Authors:** Mohamed H Yusuf, Mohammed A Alharthi, Abdulrahman S Alahmari, Gehan A Abdulaziz, Abdulaziz M Alqahtani, Fahad M Alshalfan, Yousef S Alanazi, Saeed M Alamri, Amal A Hawsawi, Rania A Alshaier, Assail N Almalki, Ahmed S Thabet, Aeyd J Alhashim, Ammar M Salawati, Faisal Al-Hawaj

**Affiliations:** 1 General Surgery, Salmaniya Medical Complex, Manama, BHR; 2 College of Medicine, King Abdulaziz University, Jeddah, SAU; 3 College of Medicine, King Khalid University, Abha, SAU; 4 College of Medicine, Taif University, Taif, SAU; 5 College of Medicine, Imam Mohammad Ibn Saud Islamic University, Riyadh, SAU; 6 College of Medicine, Jordan University of Science and Technology, Irbid, JOR; 7 General Practice, Al Madina Specialist General Hospital, Medina, SAU; 8 College of Medicine, Umm Al-Qura University, Mecca, SAU; 9 College of Medicine, Imam Abdulrahman Bin Faisal University, Dammam, SAU

**Keywords:** diabetes mellitus, hyperglycemia, hemichorea, basal ganglia, computed tomography

## Abstract

Diabetes mellitus is a prevalent metabolic disorder that has a wide range of complications. Neurological complications are common and include stroke and peripheral neuropathy. However, hemichorea is a very rare manifestation of diabetes mellitus. Chorea can be due to primary inherited conditions or secondary to other disorders. Careful evaluation of patients with chorea is crucial since secondary chorea can be managed with the treatment of the underlying cause. We report the case of a 51-year-old man who presented to the emergency department with a two-week history of sudden involuntary and random-appearing movements of the right upper and lower extremities. These movements were non-suppressible and disappeared during sleep. Further, the movements were not associated with any neurological symptoms, including headache, dizziness, weakness, sensory deficits, or loss of consciousness. The patient had a longstanding history of hypertension and diabetes mellitus. He reported that he was not compliant with his medications. Laboratory investigation revealed a very high level of blood glucose (580 mg/dL) with associated pseudohyponatreamia (127 mEq/L). Head computed tomography scan showed increased density in right caudate nuclei and putamen with no surrounding edema or mass effect. The findings were suggestive of non-ketotic hyperglycemic hemichorea based on the clinical, laboratory, and radiological laboratory findings. The patient received insulin therapy according to sliding-scale protocol. The chorea movements gradually improved and completely disappeared after the fourth day of admission with the normalization of glucose level. In view of this, emergency medicine physicians should consider non-ketotic hyperglycemia as a potential underlying etiology of acute hemichorea.

## Introduction

Chorea is a hyperkinetic movement disorder characterized by sudden and spontaneous non-repetitive movements with a random distribution that is often referred to as a dance-like movement [1]. The prevalence of chorea is unknown due to the lack of population-based studies [2]. Chorea is the classic manifestation of Huntington's disease. However, it may be caused by a variety of structural, metabolic, autoimmune, and neurodegenerative pathologies involving the basal ganglia. Such disorders include Wilson disease, Sydenham chorea, systemic lupus erythematosus, and metastatic lesions [2]. Careful evaluation of patients with chorea is crucial to identify the possible etiology [3]. Neuroimaging studies are required to rule out any structural lesions as the underlying etiology of chorea. Further, blood investigations are essential to rule out secondary chorea [2]. These include hematological and biochemical parameters. In contrast to primary hereditary chorea, chorea due to secondary causes might improve or resolve with the treatment of the underlying condition [2,3]. Here, we report the case of a patient with acute hemichorea related to his hyperglycemia, a rare manifestation of diabetes mellitus.

## Case presentation

A 51-year-old man presented to the emergency department with a two-week history of sudden involuntary and random-appearing movements of the right upper and lower extremities. These chaotic movements lasted for a few seconds and multiple times per day. The movements occurred throughout the day, but they disappear during sleep. He cannot suppress these movements and he tried to incorporate them into a purposeful movement to reduce his embarrassment. He reported that these movements affected the quality of his life as he had limited social contact because he felt embarrassed from these movements. This is the first time for him to have such movements. The movements were not associated with any neurological symptoms, including headache, dizziness, weakness, sensory deficits, or loss of consciousness.

The patient had hypertension and diabetes mellitus for the last 25 years. He reported that he was not taking his medications because of their high cost and his fear of the adverse effects of medications. He was hospitalized three years ago for a hyperosmolar hyperglycemic syndrome that occurred in association with severe pneumonia. His surgical history was significant for laparoscopic cholecystectomy performed because of recurrent attacks of biliary colic. He was not taking any medications. He worked as a school teacher. His family history was significant for colon cancer.

Upon examination, the patient demonstrated movements consistent with right hemichorea. The vital signs included a heart rate of 92 beats per minute (bpm), a temperature of 37.5℃, a respiratory rate of 20 breaths per minute, and a blood pressure of 150/92 mmHg. Apart from the choreatic movements, the neurological examination showed no evidence of focal neurological deficits. The tone and power were normal in both the upper and lower limits. The higher mental status and speech were normal. The gait and coordination were normal with no evidence of ataxia. The cardiac examination revealed a loud S2 heart sound in keeping with systemic hypertension. No added sounds or murmurs were noted. The respiratory and abdominal examinations yielded normal findings.

The patient had basic hematological and biochemical laboratory investigations. The hemoglobin level was 14.5 g/dL, the leukocytes count was 7500/μL, and the platelets count of 380,000/μL. The blood urea nitrogen (22 mg/dL) and creatinine (1.1 mg/dL) levels were slightly elevated. The liver enzymes, including alanine transaminase (18 U/L) and aspartate transaminase (17 U/L) were within the normal limits. The glucose level was significantly elevated with the level of 580 mg/dL with associated pseudohyponatremia (127 mEq/L) with the corrected sodium level being normal (134 mEq/L). The ketone levels were not elevated. Urinalysis had normal findings.

In order to rule out any structural brain abnormalities, the patient underwent a head computed tomography scan. The scan was repeated three times as the patient had difficulty lying still. It demonstrated an increased density in right caudate nuclei and putamen with no surrounding edema or mass effect. The grey-white matter differentiation was preserved and no intracranial hemorrhage was noted. The clinical and radiological findings represented a non-ketotic hyperglycemic hemichorea (Figure 1).

**Figure 1:** Head CT scan CT: computed tomography The arrow demonstrates increased density in the right basal ganglia

The patient was admitted to the medical wards. He received insulin therapy according to sliding-scale protocol. The electrolytes levels were actively monitored. The chorea movements gradually improved and completely disappeared after the fourth day of admission with the normalization of glucose level. The patient was discharged after five days of hospitalization. He was given clear instructions on the importance of taking his medications regularly. No recurrence of the abnormal movements was reported by the patient in the follow-up visit after six months.

## Discussion

We report the case of a sudden hemichorea in a middle-aged man due to non-ketotic hyperglycemia, which is a very rare manifestation of diabetes mellitus [4]. Neurological complications of diabetes mellitus, such as peripheral neuropathy and stroke, are common. However, hemichorea is a rare complication seen in less than 1 per 1,000,000 patients with diabetes mellitus [5]. In addition, chorea associated with non-ketotic hyperglycemia usually occurs in the elderly, women, and Asian ethnicity people [4]. The first case of non-ketotic hyperglycemia hemichorea was first described by Bedwell et al. in 1960 [6].

The acute onset of hemichorea is suggestive of a focal lesion in the basal ganglia. Ischemic stroke represents the most frequent cause of acute hemichorea [4]. The lesion is typically located in the contralateral side of the basal ganglia of the hemichorea. In our case, the occurrence of right hemichorea along with focal lesion in the right basal ganglia is very interesting. This has been reported previously in a few cases only [7-9]. However, an important limitation of our report is that the magnetic resonance imaging of the brain was not performed to exclude subtle contralateral basal ganglia lesions.

Non-ketotic hyperglycemia hemichorea is a rare syndrome characterized by the triad of chorea, hyperglycemia, and basal ganglia lesion [6]. The exact pathogenesis of this syndrome is unclear. Several hypotheses have been proposed to provide an explanation for this condition. It is assumed that the high glucose levels alter the autoregulatory mechanisms resulting in decreased cerebral blood flow and depletion of the gamma-aminobutyric acid (GABA) levels in the basal ganglia because of the activation of anaerobic metabolism. The reduction in the GABA, the primary inhibitory neurotransmitter in the brain, causes the non-inhibition of the excitatory neuronal signals [5,10]. Further, hyperglycemia results in impairment in the blood-brain barrier because of the high viscosity in the blood [4].

Blood glucose control is the most important treatment for non-ketotic hyperglycemia hemichorea [10]. This results in significant improvement of the hemichorea or event complete resolution. Some patients may require medical treatment (e.g., haloperidol) or surgical intervention (i.e., ventral lateral thalamotomy) if their symptoms persisted or recurred [4].

## Conclusions

Hemichorea is an extremely rare complication of diabetes mellitus. Despite this, emergency medicine physicians should remember non-ketotic hyperglycemia as a potential underlying etiology of acute hemichorea. The presented case demonstrated a rare and interesting finding of hemichorea occurring with ipsilateral basal ganglia lesion. Blood glucose control is usually a sufficient treatment for non-ketotic hyperglycemia hemichorea.
